The article "Method for Quantum Denoisers Using Convolutional Neural Network" was retracted in 2023. Reasons: unreliable results or conclusions; concerns about the data; concerns about the peer review; concerns about the citations.

# Method for Quantum Denoisers Using Convolutional Neural Network

**DOI:** 10.1155/2022/4885897

**Published:** 2022-10-06

**Authors:** Bong-Hyun Kim, S. Madhavi

**Affiliations:** ^1^School of Software, Computer Engineering Major, Seowon University 377-3, Musimseo-ro, Seowon-gu, Cheongju-si, Chungcheongbuk-do 28674, Republic of Korea; ^2^Computer Science and Engineering Department, PVP Siddhartha Institute of Technology, Kanuru, Andhra Pradesh, India

## Abstract

In many applications of quantum information science, high-dimensional entanglement is needed. Quantum teleportation is used for transferring information from one place to another using Einstein–Podolsk–Rosen pairs (EPR) and two classical bits of communication in a channel. Since we cannot produce multiple copies of an unknown state for amplification, we will generate multiple EPR pairs. However, after the distribution of the EPR pairs, they will have decreased fidelity with the ideal EPR state. So, to maintain the quantum states and maximize the quantification of the entanglement without losing the strength of the states, we propose to denoise the channel for a few types of noise. We created a random noise source and filtered out the irrelevant information without affecting the relevant information encoded in the quantum states. The proposed model is used for successful denoising of GHZ states from spin flips and bit flip errors. Much of the research work is not carried out by using machine-language-based neural networks for noise-reduction in quantum channels. In this paper, we propose a denoiser called quantum denoiser CNQD, which uses a feedforward convolution neural network model. We tuned our model with highly entangled GHZ states with zero phases and phase between [0, ∏] mixed with different kinds of noise. Finally, the proposed model can be used for optimal quantum communication via noisy quantum channels using GHZ states.

## 1. Introduction

Data aggregation is the process of aggregating data to the central node by using one or more intermediate neighbors. Some of the application areas for quantum information processing are teleportation, super-dense coding, quantum cryptography, and distant entanglement. In long-distance quantum communication, highly entangled and mixed quantum states are used. Quantum teleportation is a technique used to transfer information from one particle to another remote particle using quantum entanglement. A mixed state is said to be entangled if it cannot be represented as a mixture of un-entangled pure states.

The areas of research in entanglement are as follows:

  How to quantify entanglement in quantum states?
  How to compare entanglement in quantum states?
  How well entanglement in a quantum state is maintained through quantum channels?
  How well entanglement is preserved through quantum channels?

The article "Method for Quantum Denoisers Using Convolutional Neural Network" was retracted in 2023. Reasons: unreliable results or conclusions; concerns about the data; concerns about the peer review; concerns about the citations.

By measuring entanglement using entanglement of formation, concurrence, entanglement of distillation, relative entropy of entanglement, and negativity, we can address the first two areas, and through measuring the entanglement fidelity, the last two areas can be addressed.

Generally speaking, a quantum system cannot be fully isolated from its transmitted environment. The environment induces decoherence in the system, thereby inducing uncontrolled errors in the communication channel. Generally, nonlinear operations are required in implementing the error-correcting codes, which reduces the efficiency of the optical communication channel. Hence, quantifying the entanglement in a quantum channel is a complicated task since noise limits the efficiency of any data communication protocols.

Designing a denoising protocol is very difficult since there are many sources for noise. The noise present in the channel corrupts the state of the particle-like bit flips or may change the phase of the bit. If the channel is noisy, then the receiver will get a maximally mixed quantum state, and the measurement of such an output is completely deterministic. However, if the quantum channel is noiseless, then the encoded information can be recovered with probability 1. However, noisy channels modify the information, and the receiver obtains erroneous data.

For distant entanglement, at first, local entangled state is produced and then transmitted to a distant location using a quantum channel. Let there be two systems, *A* and *B*. Then, the local measurement is done on these two systems separately, and it satisfies the completeness relations.

(1) $$\begin{array}{c} \underset{i}{\sum }A_{i}^{+}A_{i}=I,\\ \underset{j}{\sum }B_{j}^{+}B_{j}=I,\\ \underset{ij}{\sum }A_{i}⊗B_{j}. \end{array}$$

Moreover, the joint action of systems is

(2) ρAB⟶∑iAi⊗BρABiAi+⊗Bi+.

Entanglement verification is done to specify with certainty whether a prepared state is entangled or not. Quantifying entanglement describes how much entanglement is there in a given system. Also, we can compare two systems based on the amount of entanglement in the particles that exist in the respective system. The highest entanglement indicates that the states are in their purest state. Optimal entanglement cost decreases the transmission cost of a system. The cost of entanglement cost is defined as the cost of preparing a large number *n* of copies of a given bipartite “pure” |*ϕ*_*AB*_〉|*ϕ*_*AB*_〉 states using only local operations and classical communication. If we call kmin the minimum number of EPR pairs necessary to accomplish this task, we have the entanglement cost as the limiting ratio kmin/*n*, for *n* ⟶ ∞. Minimizing the entanglement cost is the main objective for increasing any communication channel's efficiency. Similarly, distillable entanglement [1, 2] is defined as follows.

The article "Method for Quantum Denoisers Using Convolutional Neural Network" was retracted in 2023. Reasons: unreliable results or conclusions; concerns about the data; concerns about the peer review; concerns about the citations.

If *k*'max denotes the maximum number of EPR pairs that can be obtained, then we have the following:

  Distillable entanglement = ratio kmax/*n* in limit *n* ⟶ ∞.

The quantum channel acts as a medium for transferring particles between two parties. The presence of noise in the channel alters the state of the particles, like flipping the bits/changing the phase of the bit/spinning the particles, etc. Depending on the intensity of the noise levels, an original pure quantum state can be transferred into a mixed quantum state. The quantum information transmission system consists of an input quantum bit and its interaction with the environment.

Let us assume that Alice had sent a set of encoded states in a transmission channel. These encoded states reach, say, the receiver Bob. If the channel is noiseless, then the probability that Bob detects them is higher and the cost of transmission will be less. But if the channel is noisy, then Bob discards the states and both Alice and Bob repeat the process. Especially in long-distance communication, quantum entanglement plays a major role in a successful transmission.

Hence, there should be a denoiser that detects noisy states and converts them into noiseless states. The performance of a transmission channel depends on how well the denoiser performs.

The model is trained with various types of bit flip and spin flip errors during the training phase. Now, during the testing phase, the model is tested to see if it can identify the noisy states or not. The proposed model denoises the noise in the channel.

We measured the fidelity that is the probability that the denoiser is able to identify the given noisy state as a noisy state.

On a noiseless channel, the information sent by the sender can be decoded by the receiver with a probability of 1.

Generally, the probability to obtain an outcome |*j*> is defined as

(3) $$\begin{array}{c} \mathrm{Pr}\;\left(j|i\right)=Tr\left(M_{j}U\rho_{i}U^{+}\right)\text{,} \end{array}$$

where *ρ*_*i*_ denotes the density matrix for an arbitrary input state, *U* denotes an ideal unitary transformation, and *M*_*j*_ is a measurement operator.

If ^ denotes the noisy quantum process, then

(4) $$\begin{array}{c} \hat{\mathrm{Pr}}\left(j|i\right)=Tr\left(M_{j}\wedge \left(\rho_{i}\right)\right). \end{array}$$

Then, error can be quantified as follows.

The lesser the difference between $\overset{ˆ}{P}\left(j|i\right)$ and *P*(*j|i*), the higher will be the fidelity. If the fidelity is maximized, then the performance of the transmission channel is increased since the transmission cost is decreased.

The article "Method for Quantum Denoisers Using Convolutional Neural Network" was retracted in 2023. Reasons: unreliable results or conclusions; concerns about the data; concerns about the peer review; concerns about the citations.

Hence, by quantifying the errors and removing them from the encoded data, the highest entanglement can be achieved. The strength of the procedures using machine learning for noise reduction lies in the collection of training data, hyperparameter value, and simulation system size.

Section 2 discusses the literature study.  Section 3 presents the proposed algorithm for denoising the quantum commutation channel using a convolution neural network and applying the machine learning algorithm for maximizing the entanglement of the transferred data in a quantum channel.  Section 4 presents the simulation setup and results.  Section 5 presents the discussion, the limitations of the current study, and its future scope.

## 2. Related Studies

In [3], the authors studied various noise-adaptive compilermappings for noisy intermediate-scale quantum computers. After travelling a certain distance, repeaters are required to strengthen the data. Much of the research is carried out on how to overcome the limitations of such repeaters during the long-distance communications. Many machine learning algorithms are proposed to provide a method to enable the channel to understand the noise and remove it from the data. In [4], the authors studied the fundamental limits of repeater-less quantum communications and implemented a method for removing noise from the channel for improving the communication channel's efficiency. In [5], the authors studied the noise robustness of quantum neural networks. In [6], quantum variational autoencoders are proposed to remove the noise in the channel. Their implementation results are helpful for using quantum computers to train quantum variational autoencoders to obtain performance for generative models [6]. Much research is carried out for the experimental realization of a quantum autoencoder [7]. In [7], the authors implemented an autoencoder which reduces qutrits to qubits with low error levels. In [8], the authors studied a universal training algorithm for quantum deep learning. They introduced backwards quantum propagation of the phase errors principle and constructed multiple universal optimization heuristics for training deep neural networks on a quantum computer.

In [9], the authors studied quantum neuron applications in machine learning methods for noise removal. In [10], the authors studied the two aspects of quantum neural machine learning: backpropagation and dynamics. They proposed a novel quantum machine learning framework where network processing is divided into the learning stage and the backpropagation stage, where the network effectively works as a self-programing quantum computing system [10]. In [11], the authors studied the parameterized quantum circuits as machine learning models. Their work can be implemented as an application to a variety of data-driven tasks, such as supervised learning and generative modeling. In [12], the authors studied the efficient learning for deep quantum neural networks. Entanglement quantification is essential to find out if the states are affected by noise or not. In [13], the authors studied the complementary quantum capacity of the depolarizing channel. In [14], the authors studied the dephrasure channel and super-additivity of coherent information. In [15], the authors studied the experimental detection of quantum information sharing and its quantification in quantum spin systems. In [16], the authors studied the hierarchical joint remote state preparation in a noisy environment. Quantum information processing has many applications, like quantum cryptography [17] and teleportation [18], with multiple degrees of freedom for a single photon. In [19], the authors studied the quantum teleportation of a three-qubit state using a five-qubit cluster state. In [20], the authors studied practical quantum error mitigation for near-future applications. They implemented a method for minimizing the impact of errors for near-future quantum devices that suffer from a lack of resources for full fault tolerance [20]. In [21], the authors studied how the error mitigation extends the computational reach of a noisy quantum processor.

The article "Method for Quantum Denoisers Using Convolutional Neural Network" was retracted in 2023. Reasons: unreliable results or conclusions; concerns about the data; concerns about the peer review; concerns about the citations.

Quantum information processing provides solutions in the field of computer science which cannot be solved by classical communication systems, and many new versions of capacity definitions have evolved. In [22], the authors studied the quantum dynamic capacity formula of a quantum channel. They proposed a quantum dynamic capacity formula for quantum communication and entanglement on a noisy quantum channel. In [23], the authors studied the No-go theorems for quantum resource purification. By applying the laws of quantum mechanics, they found how generic and noisy resources can be purified. In [24], the authors studied the necessary and sufficient conditions for measurements of quantum channels. They demonstrated their results by applying them to fault-tolerant quantum computational applications. In [25], the authors studied the strong-converse rates for quantum communication. The authors found whether it is possible to transmit quantum information at a rate exceeding the channel capacity or not [25]. In [26], the authors studied the unscrambling entanglement through a complex medium.

The article "Method for Quantum Denoisers Using Convolutional Neural Network" was retracted in 2023. Reasons: unreliable results or conclusions; concerns about the data; concerns about the peer review; concerns about the citations.

In [27], the authors proposed a method for unscrambling entanglement through a complex medium. In [28], the authors studied protecting entanglement from decoherence using weak measurement and quantum measurement reversal. In [29], the authors studied the experimental demonstration of decoherence suppression via quantum measurement reversal. In [30], the authors studied the foundations of quantum discord. They implemented a method to protect entanglement from decoherence and proved that their scheme makes use of the quantum measurement for actively battling against decoherence. In [31], the authors studied the quantum flags and new bounds on the quantum capacity of the depolarizing channel. In [32], the authors studied the quantum information theory. In [33], the authors studied the quantum repeaters and quantum key distribution and the impact of entanglement distillation [45] on the secret key rate. In [34], the authors studied the inside of quantum repeaters. They discussed various approaches to quantum repeaters and their expected performance and limitations. In [35], the authors studied the reverse coherent information and secret key distillation over a satellite-to-satellite free-space optics channel with eavesdropper dynamic. In [36], the authors studied secret key distillation over a pure-loss quantum wiretap channel under restricted eavesdropping. In [37], the authors studied Ground-based and Airborne telescopes. In [38], the authors studied on secret key distillation over a pure loss quantum wiretap channel under restricted eavesdropping. In [39], the authors studied entanglement sharing among quantum particles with more than two orthogonal states. Many authors discussed about delay-tolerant networks. In [40], the authors studied an efficient routing using partitive clustering algorithms in Ferry-based delay tolerant networks. Many machine learning methods are implemented in improving the efficiency of networks. In [41], the authors discussed an improved energy-efficient algorithm in wireless communication systems using the PSO method. In [42], the authors discussed the “Feed Forward Networks in Color Extended Visual Cryptography to Generate Meaningful Shares.” In [43], the authors discussed [44] “Banknote Image Defect Recognition Method Based on Convolution Neural Network.”

## 3. Proposed CNQD Noise Model

GHZ states possess maximal entanglement depth and high entanglement quantification. Hence, they are used in applications requiring long-distance communication. Due to noise, the transmitted GHZ states are altered. Hence, this paper describes a method to correct the GHZ states, which are affected by noise when transmitted through a noisy channel.

The article "Method for Quantum Denoisers Using Convolutional Neural Network" was retracted in 2023. Reasons: unreliable results or conclusions; concerns about the data; concerns about the peer review; concerns about the citations.

ML algorithms are used in different learning scenarios. The proposed paper describes a model called quantum denoiser using the convolution neural network CNQD for the task of noise recognition and removal in the GHZ states. This model consists of *M* layers. The outputs of a layer are fed as inputs to the next layer. CNQD is a feedforward neural network which is constructed from simpler parameterized maps called neurons, and the outputs of the set of neurons at one layer are fed into the next layer. The depth denotes the number of layers, and the width denotes the maximal number of neurons per layer.

The general feedforward neural network consists of an input layer, a hidden layer, and an output layer. The first layer is the input layer, and the last layer is the output layer. Generally, there exists a function *f* on the input like fv(*x*) to generate the outputs. Each layer extracts the features from the input data and sends the outputs to the next layer. The network has a bottleneck layer for filtering the irrelevant features.

Here, *N* denotes the quantum channel. *ρ* In and *ρ* out are the two states denoting the input and output states. *ρE* denotes the environment. Suppose Alice *A* transmits to Bob *B* using the environment *E*. Then, *U* the unitary operation is as follows:

(5) $$\begin{array}{c} N:U_{A⟶BE}\text{.} \end{array}$$

After transmission of the quantum data on the channel *N*, the *ρE* is as follows:

(6) $$\begin{array}{c} \rho_{E}=T_{\gamma_{B}}U\rho_{in}⊗\left|0\right.\rangle \langle 0|U^{+}\text{,} \end{array}$$

where *T* traces out the output system.

Similarly, the output of the channel is described only after tracing the channel as

(7) $$\begin{array}{c} \rho_{B}=T_{\lambda_{E}}\left(U_{A⟶BE}\left(\rho_{A}a\right)\right)=N\left(\rho_{A}\right)\text{.} \end{array}$$

The unitary operation *U* acts on all qubits at the input layer and one qubit at the output layer. The network is trained with different controllable and uncontrollable noise patterns and corresponding labels.

Generally, for pure states, the entropy of entanglement is defined as *ε*(|*ψ*〉) = *S*(*tr*_*B*_|*ψ*〉〈*ψ*|) where *S* is the entropy and *B* is a subsystem.

For mixed states, the entanglement is quantified in terms of entanglement formation for a state *ρ* and is defined as $\varepsilon_{F}\left(\rho \right)=inf\left(\underset{i}{\sum }\rho_{i}\right.S\left(tr_{B}\left|\psi_{i}\right.\rangle \langle \left.\psi_{i}\right|\right)$ where $\rho =\underset{i}{\sum }\rho_{i}\left|\psi_{i}\right.\rangle \langle \left.\psi_{i}\right|$. The entanglement cost is defined as $\varepsilon_{C}\left(\rho \right)=\lim\underset{n⟶\infty }{\varepsilon_{F}}\left(\rho^{⊗n}\right)/n$.

The article "Method for Quantum Denoisers Using Convolutional Neural Network" was retracted in 2023. Reasons: unreliable results or conclusions; concerns about the data; concerns about the peer review; concerns about the citations.

Generally, the process of information transmission through a quantum communication channel has three main steps. Alice *A* encodes her information as qubits and sends them to Bob *B* through the communication channel. Suppose the quantum channel *N* is noisy. Then, the channel mixes noise data with this encoded data. To identify whether noise is mixed in the transmission state, fidelity is calculated, through which we can determine the closeness.  Figure 1 shows the two states, that is, the states before and after the noise is mixed.

Finally, Bob *B* measures on the received data and identifies the noise. To recover the message sent by Alice *A*, Bob *B* performs data recovery steps. If there are m layers in the feedforward neural network, then

(8) $$\begin{array}{c} \begin{array}{c} N\left(\rho_{in}\right)=N^{M}\left(..\right.N^{2}\left.\left(\rho_{in}\right)\right).\left..\right)⟶11\\ N^{k}\left(\rho_{k-1}\right)\equiv tr_{k-1}\left(U\left(\rho_{k-1}⊗{\left({\left|↓\right.\rangle }_{out}\langle \left.↓\right|\right)}^{⊗m}\right)U^{+}\right) \end{array}\text{.} \end{array}$$

The cost of transmission in the channel *C* is as follows:

(9) $$\begin{array}{c} C\left(k\right)=\frac{1}{N}\sum \sum \left({\left|\Phi \right.\rangle }_{i}\right.,\rho_{i}^{k}. \end{array}$$

At the ith training state |*φ*_*i*_〉, *F* denotes the fidelity, *ρ* denotes the density matrix, *N* denotes the number of training pairs, and *K* denotes the number of parameters.

Figure 1 illustrates how the proposed model is trained to denoising the channel. Let there be *K* features in the input, and after a fixed number of steps, the proposed model minimizes the noise. In the assumed CNQD, the inputs are given at the input layer and the outputs fv(*x*) are in the last layer. If the training data consists of (*x*_*i*_,*y*_*i*_) *i* = 1 to *L* € *X*2 x *Y*2 tuned with appropriate hyper parameter, the function to minimize the cost is as follows:

(10) $$\begin{array}{c} C\left({\left\{x_{i},y_{i}\right\}}_{i=1^{L}}=\frac{1}{L}\overset{L}{\underset{i=1}{\sum }}d\left(f_{v}\left(x_{i}\right),y_{i}\right)\right). \end{array}$$

where fv(*x*_*i*_) is the output for a given label *y*_*i*_.

The training algorithm is as follows.

### 3.1. Algorithm CNQD (A, B, *E*, and *N*)

Let *N* denote the quantum channel:

 
*ρ* In and *ρ* out are the two states denoting the input and output states.
 
*ρE* denotes the environment. *U* is the unitary operation.
  Let Alice *A* transmit to Bob *B* using the environment *E*.

Fidelity measure is used to find out how much entanglement difference occurs between the two quantum states. That is, it is used to measure the probability that one state has.

The article "Method for Quantum Denoisers Using Convolutional Neural Network" was retracted in 2023. Reasons: unreliable results or conclusions; concerns about the data; concerns about the peer review; concerns about the citations.

The distance between the label *y*_*i*_ and point fv(*x*_*i*_) should be minimum such that the model is assumed to be trained perfectly to denoise the channel. The objective of the proposed model is to minimize the transmission cost by maximizing the fidelity of the transmission channel. By using a general model of a noisy quantum communication channel, we attempt to apply a fully connected quantum network to the task of reconstructing noiseless results from quantum simulation data from a noisy channel, where *x* is the input, ʘ is the learnable weights of the model, *f* (.) is the function which learns from the hidden layers of the input, and *g* (.) is the function which maps back to the values of the training examples.

Applying the principle of no-cloning denoising CNQD as shown in Figure 2 with fully connected layers, a minimized cost function is obtained. The quantum data mixed with noise is passed to the assumed model. The output will be the quantum data without noise; that is, the noise is filtered from the quantum input data.

## 4. Simulation

We simulated the CNQD protocol for denoising the bit flip and spin flip errors in the quantum channel. For a small time, *T*, let *m* qubits be assumed to be flipped at rate ℾ with a probability *ρ* in each training phase. These errors generate noise and can be simulated using Qiskit's quantum air noise simulator. The training data is { |*ψ*_*i*_〉, |*ψ*_*i*_〉 } *i* = 1..L, ∈ *H*, where *U*| is with probability 1 − *ρ* and a random pure state is sampled from a uniform distribution with probability *ρ* on the *m*-qubit GHZ.

The proposed CNQD for the m-qubit GHZ state is trained first with random bit flips with a flip probability in the range [0.1–1]. We had approximately 300 training pair which consisted of 200 pairs drawn from the affected GHZ states, and at the end of each epoch, the fidelity is calculated. Also, the average fidelity at the end of the first 90 epochs tested on the data is 0.9982 with the flip probability of 0.2.

Figure 3 shows how CNQD denoises bit flip errors. It shows the average fidelity before denoising and after denoising. Similarly, for GHZ with a zero phase spin flip errors with a probability of 0.2 average fidelity, it is 0.96 after 160 training pairs and training rounds to end up in a flipped state, with spin flip errors. Also, after 200 noisy GHZ with phases *φ* ∈ (0, *π*), the average fidelity is observed to be 0.9968 with a probability of *p* = 0.3. Figures 4 show how CNQD denoises spin flip errors with GHZ = 0 and Figure 5 show how CNQD denoises spin flip errors with GHZ = *φ* ∈ (0, *π*).

The article "Method for Quantum Denoisers Using Convolutional Neural Network" was retracted in 2023. Reasons: unreliable results or conclusions; concerns about the data; concerns about the peer review; concerns about the citations.

It shows the average fidelity before denoising and after denoising. Now the output labels consist of both known and unknown noise bits. Since the trained model successfully detected the known noise distribution, we will test the model to detect the unknown noise bits too. We tested the network model for bit flips and spin flips with phase changes for 500 rounds on a 100 noisy test set consisting of bit flip errors, spin flips with GHZ = 0, and spin flips with GHZ = *φ* ∈ (0, *π*) states, and it was found that the model is able to remove the noise with a flip probability of 0.4. Hence, the proposed model is trained successfully for the removal of noise in input data.

## 5. Discussion

We assumed a dense network with nodes spreading in an area of 200 × 200 sq units. We have simulated a method for denoising quantum channels by filtering various noises like bit flips, and spin flips with phase changes in the quantum channels by tuning the learning rate and the probability of the flip rates to different values. The results show that the proposed model can be used for any applications involving long-distance communications successfully, either with high entanglement or without being affected by noise. But along with bit flip errors and spin flip errors, the channels are prone to various types of errors. One limitation of the study is that the model identifies and denoises only two types of errors. In the future, it will be trained for other types of noises found in quantum communication channels.

## Figures and Tables

**Figure 1:** Network architecture of CNQD.

**Figure 2:** The general quantum channel with noise.

**Figure 3:** CNQD denoises bit flip errors.

**Figure 4:** CNQD denoises spin flip errors with GHZ = 0.

**Figure 5:** CNQD denoises spin flip errors with GHZ *φ* ∈ (0, *π*).

## Data Availability

No data were used to support the study.

## References

[1] Uhlmann A. (1976). The “transition probability” in the state space of a -algebra. *Reports on Mathematical Physics*.

[2] Fang K., Wang X., Tomamichel M., Duan R. (2017). Non-asymptotic entanglement distillation. https://arxiv.org/abs/1706.06221.

[3] Murali P., Baker J. M., Javadi-Abhari A., Chong F. T., Martonosi M. (2017). Noise-adaptive compiler mappings for noisy intermediate-scale quantum computers. *Proceedings of the Twenty-Fourth International Conference on Architectural Support for Programming Languages and Operating Systems*.

[4] Pirandola S., Laurenza R., Ottaviani C., Banchi L. (2017). Fundamental limits of repeaterless quantum communications. *Nature Communications*.

[5] Kalb N., Reiserer A. A., Humphreys P. C. (2017). Entanglement distillation between solid-state quantum network nodes. *Science*.

The article "Method for Quantum Denoisers Using Convolutional Neural Network" was retracted in 2023. Reasons: unreliable results or conclusions; concerns about the data; concerns about the peer review; concerns about the citations.

[6] Scheiermann D. (2019). Noise robustness of quantum neural networks. *Bachelor’s Thesis*.

[7] Khoshaman A., Vinci W., Denis B., Andriyash E., Sadeghi H., Amin M. H. (2018). Quantum variational autoencoder. *Quantum Sci. Technol.*.

[8] Pepper A., Tischler N., Pryde G. J. (2019). Experimental realization of a quantum autoencoder: the compression of qutrits via machine learning. *Physical Review Letters*.

[9] Verdon G., Pye J., Broughton M. (2018). A universal training algorithm for quantum deep learning. http://arxiv.org/abs/1806.09729.

[10] Cao Y., Guerreschi G. G., Aspuru-Guzik A. (2017). Quantum neuron: an elementary building block for machine learning on quantum computers. https://arxiv.org/abs/1711.11240.

[11] Gon calves C. P. (2017). Quantum neural machine learning: backpropagation and dynamics. *NeuroQuantology*.

[12] Benedetti M., Lloyd E., Sack S. (2019). Parameterized quantum circuits as machine learning odels. http://arxiv.org/abs/1906.07682.

[13] Beer K., Bondarenko D., Farrelly T., Osborne T. J., Salzmann R., Wolf R. (2019). E_cient learning for deep quantum neural networks.

[14] Leung D., Watrous J. (2017). On the complementary quantum capacity of the depolarizing channel. *Quantum*.

[15] Bennett C. H., Bessette F., Brassard G., Salvail L., Smolin J. (1992). Experimental quantum cryptography. *Journal of Cryptology*.

[16] Das D., Singh H., Chakraborty T., Gopal R. K., Mitra C. (2013). Experimental detection of quantum information sharing and its quantification in quantum spin systems. *New Journal of Physics*.

[17] Leditzky F., Leung D., Smith G. (2018). Dephrasure Channel and superadditivity of coherent information. *Physical Review Letters*.

[18] Shukla C., Thapliyal K., Pathak A. (2017). Hierarchical joint remote state preparation in noisy environment. *Quan-tum Inf. Process*.

[19] Wang X. L., Cai X. D., Su Z. E. (2015). Quantumteleportation of multiple degrees of freedom of a single photon. *Nature*.

[20] Liu Z. M., Zhou L. (2014). Quantum teleportation of a three-qubit state using a five-qubit cluster state. *International Journal of Theoretical Physics*.

[21] Endo S., Benjamin S. C., Li Y. (2018). Practical quantum error mitigation for near-future applications. *Physics Reviews X*.

[22] Kandala A., Temme K., Corcoles A. D., Mezzacapo A., Chow J. M., Gambetta J. M. (2019). Error mitigation extends the computational reach of a noisy quantum processor. *Nature*.

[23] Wilde M. M., Hsieh M. H. (2012). The quantum dynamic capacity formula of a quantum channel. *Quantum Information Processing*.

[24] Fang K., Liu Z.-W. (2020). No-go theorems for quantum resource purification: new approach and channel theory. http://arxiv.org/abs/2010.11822.

The article "Method for Quantum Denoisers Using Convolutional Neural Network" was retracted in 2023. Reasons: unreliable results or conclusions; concerns about the data; concerns about the peer review; concerns about the citations.

[25] Burniston J., Grabowecky M., Scandolo C. M., Chiribella G., Gour G. (2020). Necessary and sufficient conditions on measurements of quantum channels. *Proc. R. Soc. A*.

[26] Tomamichel M., Wilde M. M., Winter A. (2017). Strong converse rates for quantum communication. *IEEE Transactions on Information Theory*.

[27] Valencia N. H., Goel S., McCutcheon W., Defienne H., Malik M. (2020). Unscrambling entanglement through a complex medium. *Nature Physics*.

[28] Lee J.-C., Jeong Y.-C., Kim Y.-S., Kim Y.-H. (2011). Experimental demonstration of decoherence suppression via quantum measurement reversal. *Optics Express*.

[29] Kim Y.-S., Lee J.-C., Kwon O., Kim Y.-H. (2012). Protecting entanglement from decoherence using weak measurement and quantum measurement reversal. *Nature Physics*.

[30] Vedral V. (2017). *Foundations of Quantum Discord Lectures on General Quantum Correlations and Their Applications*.

[31] Fanizza M., Kianvash F., Giovannetti V. (2020). Quantum flags and new bounds on the quantum capacity of the depolarizing channel. *Physical Review Letters*.

[32] Wilde M. M. (2017). *Quantum Information Theory*.

[33] Bratzik S., Abruzzo S., Kampermann H., Bruß D. (2013). Quantum repeaters and quantum key distribution: the impact of entanglement distillation on the secret key rate. *Physical Review A*.

[34] Munro W. J., Azuma K., Tamaki K., Nemoto K. (2015). Inside quantum repeaters. Selected topics in quantum electronics. *IEEE Journal of*.

[35] Garca-Patron R., Pirandola S., Lloyd S., Shapiro J. H. (2009). Reverse coherent information. *Physical Review Letters*.

[36] Pan Z., Djordjevic I. B. (2012). Secret key distillation over satellite-to-satellite free-space Optics Channel with eaves dropper dynamic positioning. http://arxiv.org/abs/2012.13865.

[37] Johns M., McCarthy P., Raybould K. (2012). Giant magellan . Telescope overview. *Ground-Based and Airborne Telescopes IV*.

[38] Pan Z., Seshadreesan K. P., Clark W. Secret key distillation over a pure loss quantum wiretap channel under restricted eavesdropping.

[39] Dennison K. A., Wootters W. K. (2001). Entanglement sharing among quantum particles with more than two orthogonal states. *Physics Reviews*.

[40] Benenti G., Casati G., Strini G. (2007). *Principles of Quantum Computation and Information - Volume II: Basic Tools*.

[41] Jedari B., Goudarzi R., Dehghan M. (2009). Efficient routing using partitive clustering algorithms in ferry-based delay tolerant networks. *International Journal of Future Generation Communication and Networking, NADIA, ISSN*.

[42] Achki S., Gharnati F. (2017). Improved energy-efficient algorithm in wireless communication systems using PSO method. *International Journal of Future Generation Communication and Networking*.

The article "Method for Quantum Denoisers Using Convolutional Neural Network" was retracted in 2023. Reasons: unreliable results or conclusions; concerns about the data; concerns about the peer review; concerns about the citations.

[43] Ida Christy J., Seenivasagam V. (2015). Feed forward networks in color extended visual cryptography to generate meaningful shares. *International Journal of Security and Its Applications*.

[44] Wang K., Wang H., Yue S., Li M., Qiu F. (2016). Banknote image Defect recognition method based on convolution neural network. *International Journal of Security and Its Applications*.

[45] Rozpędek F., Schiet T., . L. P, Elkouss D., Doherty A. C., Wehner S. (2018). Optimizing practical entanglement distillation. *Physics Reviews*.

